# The Establishment of a Mouse Model for Degenerative Kyphoscoliosis Based on Senescence-Accelerated Mouse Prone 8

This article has been retracted.

**DOI:** 10.1155/2022/7378403

**Published:** 2022-07-20

**Authors:** Zongshan Hu, Ziyang Tang, Abdukahar Kiram, Jie Li, Hui Xu, Yanjie Xu, Huiming Jiang, Zezhang Zhu, Yong Qiu, Zhen Liu

**Affiliations:** ^1^Division of Spine Surgery, Department of Orthopedic Surgery, Nanjing Drum Tower Hospital, The Affiliated Hospital of Nanjing University Medical School, China; ^2^Division of Spine Surgery, Department of Orthopedic Surgery, Nanjing Drum Tower Hospital, The Clinical College of Nanjing Medical University, China

## Abstract

**Objective:**

Degenerative kyphoscoliosis (DKS) is a complex spinal deformity associated with degeneration of bones, muscles, discs, and facet joints. The aim of this study was to establish an animal model of degenerative scoliosis that recapitulates key pathological features of DKS and to validate the degenerative changes in senescence-accelerated mouse prone 8 (SAMP8) mice.

**Methods:**

Thirty male mice were divided into 2 groups: 10 bipedal C57BL/6J mice were used as the control group, and 20 bipedal SAMP8 mice were used as the experimental group. Mice were bipedalized under general anesthesia. The incidence of scoliosis and bone quality was determined using radiographs and in vivo micro-CT images 4, 8, and 12 weeks after surgery, respectively. Histomorphological studies of muscle samples were performed after sacrifice at 12 weeks after surgery.

**Results:**

On the 12th week, the incidence rates of kyphosis in C57BL/6J and SAMP8 groups were 50% and 100%, respectively. Overall, the incidence and angle of kyphosis were significantly higher in the bipedal SAMP8 group compared to the C57BL/6J group (44.7°± 6.2° vs. 84.3°± 10.3°, P<0.001). Based on 3D reconstruction of the entire spine, degeneration of the intervertebral disc was observed in bipedal SAMP8 mice, including the reduction of disc height and the formation of vertebral osteophytes. The bone volume ratio (BV/TV) was significantly suppressed in the bipedal SAMP8 group compared with the bipedal C57BL/6J group. In addition, HE staining and Mason staining of the paraspinal muscle tissue showed chronic inflammation and fibrosis in the muscles of the bipedal SAMP8 group.

**Conclusions:**

The SAMP8 mouse model can be taken as a clinically relevant model of DKS, and accelerated aging of the musculoskeletal system promotes the development of kyphosis.

## 1. Introduction

Degenerative kyphoscoliosis (DKS) is a coronal deviation of the spine, prevalent in the elderly. Most DKS cases occur in the lumbar segment of the spine (the Cobb angle of the coronal plane > 10°) [1, 2]. DKS involves progressive and asymmetric degeneration of the intervertebral discs, facet joints, and other structural spinal components, often resulting in nerve compression [3]. The reported incidence of DKS was 0.087%, and the median age was 64.9 ± 9.4 years. The incidence is significantly higher in older women than in older men [4, 5]. With the gradual aging of the population, DKS seriously affects the quality of life of the elderly and poses a threat to the life of the elderly [6].

With the increase in DKS patients, in order to better understand the pathogenesis of DKS, animal models of scoliosis have been established using different animals, such as Sprague-Dawley (SD) rats [7], pigs [8], goats [9], C57BL/6 mice [10], and baboons [11]. A mouse model of DKS using heparin has also been recently reported. Heparin increased the incidence of scoliosis in C57BL/6J biped mice and resulted in more severe deformity in a relatively short period of time [12]. The occurrence of DKS is age-related. It is common in middle-aged and elderly people. The mean age of the patients was approximately 60 years [13]. The accelerated aging mouse (SAM) established by Takahashi is the only mammalian model currently used to study accelerated aging. These mammals include SAMP1, SAMP6, SAMP8, SAMP10, SAMR1, and others [14]. SAMP1 mice are commonly used to study animal models of senile amyloidosis [15]. SAMP6 mice have been developed as a spontaneous experimental model of senile osteoporosis [16]. SAMP8 mice are a model for studying the effects of aging on cardiovascular health [17] and neurodegenerative diseases [18]. Notably, SAMP8 mice are frequently used to study neurodegenerative diseases, but they can also be used to study degenerative joint diseases [19]. Studies have shown that SAMP8 mice may simultaneously develop sarcopenia, osteoporotic fractures, and other symptoms [20]. Sarcopenia affects muscle performance and is considered a major cause of functional limitation and exercise dependence in older adults with osteoporosis [21]. Osteoporosis is a cause of DKS. However, the association between sarcopenia, osteoporosis, and DKS remains unclear, in part due to the lack of relevant animal models to study. Therefore, in this study, we aimed to construct an animal model of DKS through SAMP8 mice and to explore the relevant clinical manifestations of the model animals of DKS.

## 2. Materials and Methods

### 2.1. Animal

Adult male C57BL/6J mice (*N* = 10, 10-12 weeks old, 20-24 g body weight) and male SAMP8 mice (*N* = 20, 20-21 weeks old, 22-25 g body weight) were obtained from Nanjing University Medicine obtained from the Animal Experiment Center of the Chinese Academy of Sciences. Animals were housed under standard conditions (12 h light/dark cycle, 22-25°C, 50% relative humidity) with free access to food and water. The protocol of animal experiments has been approved by the Animal Care Committee of Nanjing University School of Medicine (approval number MSNU20210013), and the animal experiments were carried out in accordance with the National Institutes of Health Guidelines for the Care and Use of Laboratory Animals.

### 2.2. The Construction of the Bipedal Upright Model

C57BL/6J and SAMP8 mice were anesthetized by intraperitoneal injection of 3% sodium phenobarbital (30 mg/kg). After anesthesia, the skin of the mice was incised in the supine position at the level of the scapulae of both forelimbs. Both forelimbs were securely ligated with silk thread above the proximal skin edge. Then, the distal limb is excised, and the bleeding is appropriately stopped. The skin is sutured, and the stump is buried. The tail was firmly ligated and then removed. Finally, a bipedal mouse model was constructed. After surgery, animals are housed in specially designed cages to recover for 3 to 5 days. In the cage, the mice had to stand up to feed and remain standing for 2 weeks. Monthly, X-rays of the entire spine were performed. Twelve weeks later, mice were anesthetized with 3% sodium phenobarbital (30 mg/kg) and sacrificed and underwent X-ray, micro-CT, and histological examinations (Figure 1).

### 2.3. X-Ray Examination

Twelve weeks after surgery, mice were placed supine on a camera table under anesthesia. Take anterior, posterior, and lateral radiographs of the animal. Observe the spine curve. Spinal curvature was measured by the Cobb method (Cobb > 10° represents scoliosis). The Cobb angle of each group of mice was measured.

### 2.4. Micro-CT

Twelve weeks after surgery, mice were anesthetized with 3% sodium phenobarbital intraperitoneally. The spines of mice were harvested, and the continuity and integrity of the spines were maintained. The soft tissue surrounding the spine was removed and fixed in 4% paraformaldehyde for 24 h. The ratio of bone volume to total volume (BV/TV, %) was examined using micro-CT (Belgium Skyscan, Skyscan-1076) and scanned with 50 kV and 200 *μ*A settings and a 0.5 mm aluminum filter. Resolution is adjusted to 26.6 microns per pixel. Each rotation step is 0.70 degrees over a range of 180 degrees. The binarized 3D image was generated with CTVox (version 2.4) [22].

### 2.5. H&E Staining

Mice were anesthetized by intraperitoneal injection of 3% sodium phenobarbital. After anesthesia, mice were sacrificed by cervical dislocation. The paraspinal muscle tissue of mice in each group was taken and fixed in formalin for 1 day. Tissues were embedded in paraffin, sliced (4 *μ*m thick), and baked in a constant temperature oven (65°C) for 6 h. Sections were routinely dewaxed, hydrated, stained with H&E, sealed with neutral glue, and observed under a microscope (Leica, Germany).

### 2.6. Masson Staining

Collagen fibers and muscle fibers in mouse paraspinal muscle tissue were examined using a Masson staining kit (Solarbio, Beijing, China) according to the manufacturer's protocol. The morphology of each slice was observed using a Leica DMI6000 B microscope (Leica, Germany).

### 2.7. Statistical Analysis

Statistical analysis was performed using SPSS 17.0 software (SPSS Inc., Chicago, IL, USA). Measurement data are expressed as mean ± standard deviation (SD). Differences between two groups were compared by the independent *t*-test, and differences among multiple groups were compared by one-way ANOVA. *P* < 0.05 was considered statistically significant.

## 3. Results

### 3.1. The X-Ray Examination and Micro-CT Evaluation of Spinal Deformities in SAMP8 Mice

We constructed C57BL/6J and SAMP8 mouse DKS models, respectively. After twelve weeks, the mice were assessed for scoliosis by X-ray. The results showed that 50% of C57 mice developed kyphosis with an angle of 44.7° ± 6.2. All SAMP8 mice developed kyphosis with a Cobb angle of 84.3° ± 10.3°. Overall, the incidence of kyphosis was higher in the SAMP8 group than in the C57 group (Figure 2(a), *P* < 0.001). Spinal deformities were further investigated using micro-CT. 3D reconstruction images showed that SAMP8 mice exhibited more severe kyphosis, decreased intervertebral height, and vertebral osteophyte formation. The bone volume ratio (BV/TV) of the SAMP8 group was significantly lower than that of the C57 group (Figures 2(b) and 2(c), *P* < 0.001).

### 3.2. The Histological Changes of SAMP8 Mice

Inflammation and muscle fibrosis in paraspinal muscle tissue of C57BL/6J and SAMP8 mice were examined by HE staining and Masson staining. HE staining showed that adipocytes and inflammatory cells were more concentrated in the muscle tissue of SAMP8 mice compared with C57BL/6J mice. Masson staining showed that the area of adipose and fibrotic tissue increased in the paraspinal muscle tissue of SAMP8 mice, suggesting significant chronic inflammation and fibrosis in their muscles (Figure 3).

## 4. Discussion

The lateral deviation of the spine usually occurs after age 50. As the population ages, the incidence of DKS also increases [2, 23]. The etiology of the disease remains poorly understood, but the most common causes include osteoporosis and degenerative disc disease [24]. Surgery is currently the most common strategy for the treatment of DKS. However, surgery is indicated for patients with moderate symptoms, large or progressive deformity, moderate spinal or foraminal stenosis, or sagittal imbalance. It is not suitable for patients with mild symptoms and less stable deformity but without sagittal imbalance or moderate stenosis, especially in elderly patients with multiple complications [25]. Therefore, establishing a suitable animal model will lay the foundation for studying the pathogenesis and treatment strategies of DKS. In this study, we used SAMP8 mice to establish a bipedal erection model. Our results showed that the incidence and angle of kyphosis were significantly higher in the bipedal SAMP8 group than in the C57BL/6J group, suggesting that the SAMP8 mouse model can be used as a clinical research model for DKS.

The SAM model was first established in 1981 and includes 9 major SAMP subtypes and 3 major aging-accelerated mouse resistance (SAMR) subtypes. Each subtype exhibits characteristic symptoms. Recently, SAMP8 mice have attracted the attention of gerontological studies due to their characteristic learning and memory impairment in old age [26]. SAMP8 mice are widely used in the study of aging-related diseases such as AD [27], cardiovascular disease [28], and age-related hearing loss [29]. More importantly, when SAMP8 mice underwent ovariectomy (OVX-SAMP8) 4 months after birth, osteoporosis was rapidly induced and bone mineral content was greatly reduced [30]. However, this study only focused on female mice, and secondary osteoporosis is caused by a lack of estrogen. Myofibrillar protein was significantly attenuated in skeletal muscle of SAMP8 mice compared to control SAMR1 mice [31, 32]. DKS usually occurs in elderly patients. Sarcopenia and osteoporosis are significantly associated with DKS [33, 34]. Therefore, SAMP8 mice can better mimic the development of DKS.

X-ray and micro-CT can be used for the diagnosis of DKS in clinical practice. In the case of osteoporosis and intervertebral disc degeneration, the morphological changes determined by X-ray are very important for the judgment of the diagnosis. Therefore, X-rays cannot be replaced by bone mineral measurements, CT, MR, or other imaging techniques. Micro-CT is a nondestructive 3D imaging technique that can generate nondestructive 3D images of trabecular bone microstructure, demonstrate the microstructure of trabecular bone, and determine bone parameters. The X-ray films are reflected in the scoliosis model established using FGFR3-/- mice; the spines of FGFR3-/- mice showed a clear curve and a larger Cobb angle. Micro-CT showed sparse pyramidal foramen structure, decreased BV/TV ratio, and significantly increased vertebral body length in FGFR3-/- mice [35]. Here, we harvested the entire spine of the mice following 12-week modeling. X-ray films suggested that 50% of C57 mice developed kyphosis with an angle of 44.7° ± 6.2, and 100% of SAMP8 mice manifested kyphosis with a Cobb angle of 84.3° ± 10.3°. Micro-CT further examined spinal deformities. 3D reconstructed images displayed that the kyphosis of SAMP8 mice was much more severe, and the BV/TV ratio of the SAMP8 group was considerably lower than that of C57 group. All these findings demonstrated that we successfully established a DKS mouse model in SAMP8 mice by making them stand upright on two feet.

The muscles that attach to the spine, the paraspinal muscles, play a vital role in maintaining the function of the spine and the entire body. Spinal lesions can directly lead to changes in the structure and function of the paraspinal muscles. Alterations in muscle structure and function, especially fatty infiltration and fibrosis, are clearly associated with spinal disorders [36]. An increasing number of studies have shown that in patients with DKS, the cross-sectional area of the lumbar erector spinae and psoas major is significantly thinner, and pathological assessment shows muscle atrophy, necrosis, and hyaline fibrosis, while muscle fat infiltration and inflammatory cell infiltration are more pronounced [37–39]. Therefore, we also performed pathological examination of the paraspinal muscle tissue of DKS mice by HE staining and Masson staining. The results showed an increase in adipocytes and inflammatory cells in the muscle tissue of SAMP8 mice. Masson staining showed that the area of adipose and fibrotic tissue in the paraspinal muscle tissue of SAMP8 mice was enlarged, indicating obvious muscle fibrosis. These findings further confirm the reliability of the DKS model using SAMP8 mice.

## 5. Conclusion

In conclusion, we successfully established an animal model of DKS using SAMP8 mice. X-ray films, micro-CT, and related histological examinations confirmed the validity of the model. We provide a reliable animal model for further study of DKS. However, the number of mouse samples in our study was not sufficient. Therefore, we will increase our sample in the next study to further confirm the validity of the DKS model using SAMP8 mice.

## Figures and Tables

**Figure 1:** The schematic diagrams of experimental designs.

**Figure 2:** X-ray and micro-CT assessment of spinal deformities in SAMP8 mice. (a) X-ray examination of mouse spine morphology and calculation of mouse Cobb angle. ^∗^*P* < 0.001, *n* = 10/group. (b, c) Micro-CT was used to assess trabecular bone microstructure in mice by 3D imaging and to measure the bone volume ratio (BV/TV). ^∗^*P* < 0.001, *n* = 8/group.

**Figure 3:** Histological changes in SAMP8 mice. (a) HE staining to examine chronic adipose proliferation in mouse paraspinal muscle tissue. (b) Masson staining to measure collagen fibers and muscle fibers in paraspinal muscle tissue in mice. Scale = 50 *μ*m.

## Data Availability

All data were included in the manuscript.
